# A CAD System for Alzheimer's Disease Classification Using Neuroimaging MRI 2D Slices

**DOI:** 10.1155/2022/8680737

**Published:** 2022-08-09

**Authors:** Monika Sethi, Shalli Rani, Aman Singh, Juan Luis Vidal Mazón

**Affiliations:** ^1^Chitkara University Institute of Engineering & Technology, Chitkara University, Punjab, India; ^2^Faculty of Engineering, Universidade Internacional do Cuanza, Estrada Nacional 250, Bairro Kaluapanda, Cuito-Bié, Angola; ^3^Higher Polytechnic School, Universidad Europea del Atlántico, C/Isabel Torres 21, 39011 Santander, Spain; ^4^Department of Project Management, Universidad Internacional Iberoamericana, Campeche 24560, Mexico

## Abstract

Developments in medical care have inspired wide interest in the current decade, especially to their services to individuals living prolonged and healthier lives. Alzheimer's disease (AD) is the most chronic neurodegeneration and dementia-causing disorder. Economic expense of treating AD patients is expected to grow. The requirement of developing a computer-aided technique for early AD categorization becomes even more essential. Deep learning (DL) models offer numerous benefits against machine learning tools. Several latest experiments that exploited brain magnetic resonance imaging (MRI) scans and convolutional neural networks (CNN) for AD classification showed promising conclusions. CNN's receptive field aids in the extraction of main recognizable features from these MRI scans. In order to increase classification accuracy, a new adaptive model based on CNN and support vector machines (SVM) is presented in the research, combining both the CNN's capabilities in feature extraction and SVM in classification. The objective of this research is to build a hybrid CNN-SVM model for classifying AD using the MRI ADNI dataset. Experimental results reveal that the hybrid CNN-SVM model outperforms the CNN model alone, with relative improvements of 3.4%, 1.09%, 0.85%, and 2.82% on the testing dataset for AD vs. cognitive normal (CN), CN vs. mild cognitive impairment (MCI), AD vs. MCI, and CN vs. MCI vs. AD, respectively. Finally, the proposed approach has been further experimented on OASIS dataset leading to accuracy of 86.2%.

## 1. Introduction

Healthcare problems are by far the most widely discussed subjects in the worldwide, so both healthcare providers and academics are working constantly to advance clinical diagnosis, therapies, and assessments aimed at saving sufferer's lives and improve healthy living. AD is one of the medical disorders that are posing a threat to human health [1]. AD and cerebrovascular disorder are two major types of dementia. Dementia is a neurological brains condition defined by continual declining cognitive abilities [2]. For the moment, there is no cure for AD, and it is considered destructive to individual life and vitality. Many individuals all across the world have been impacted by it. According to the statistics in [3], AD is the 6th leading cause of mortality in the United States, and the 5th leading cause of death in older adults above the age of 65. Although several other causes of mortality have all been falling, fatality rate from AD has been tremendously rising. Around 2000 to 2006, fatality from heart complications lowered by roughly 12%, blood clot mortality declined by 18%, and prostatic cancer-related casualties dropped by 14%; however, mortality from AD rose by 47%. On the other hand, lives lost from AD grew by 89% as per the reports in [4]. According to estimates regarding AD in 2019 Alzheimer's disease facts and figures, the number of individuals lost from AD will be quadrupled by 2050.The exact count of deaths caused by AD is probably much higher than documented on official records. An approximately 18.5 billion hours of assistance were given to persons having AD or other brain disorders by more than 16 million close relatives in 2018 [5]. AD-related neuroanatomical biomarkers are researched several years prior clinical features of cognitive problems, meaning that AD progression might well be identified in vivo biomarker analysis [6, 7]. Biomarkers include positron emission tomography (PET), MRI, and blood or cerebrospinal fluid. MRI is widely employed in the identification and diagnosis of AD. MRI scans have numerous benefits over the comparative techniques. For instance, it does not utilize radiation exposure and therefore is noninvasive, cheaper, and even more readily available in clinical settings. Furthermore, MRI indicators could collect heterogeneous information during the same imaging sessions [8]. The visual examination, on the other hand, is prone to human visual constraints and several other factors such as judgment and the clinician's expertise [9]. Furthermore, the health sector acts as a set of independent units, such as clinics, industrial, and healthcare departments. As a result, increased data exchange across such institutions is required to better understand the symptoms, any new evolutions, and the related test findings [10–12].

On the other hand, various machine learning (ML) algorithms applied to structural MRI have been employed in past studies to classify AD individuals against to normal healthy people. One of most widely used ML approach is the support vector machine (SVM) [13]. This technique extricates high-dimensional, meaningful features from MRI scans to develop classifier which automates the diagnosis of AD. ML classification comprises of two main steps, namely, feature engineering (feature extrication+feature selection and then dimensionality reduction), and based on those features, lastly classification takes place. Such approach has several limitations as it demands extensive data preprocessing, which requires a lot of time and involves massive mathematics [14, 15]. Additionally, the scalability from these techniques is regarded as a crucial problem [16]. DL techniques have significant benefits over traditional ML approaches [17]. Moreover, neural networks are being used in artificial intelligence systems [18]. For instance, such techniques need not involve image preprocessing and therefore can acquire appropriate features from raw imaging data without human intervention. One such result in methods, those are less labor intensive, unbiased, and highly objective. DL methods as previously discussed are ideally suited to managing large, high-dimensional medical image processing. As per experimental research, CNN, a DL technique, outperforms conventional ML algorithms.

AD is indeed an incurable neurological disorder that causes gradual mental decline, often in the elderly. The purpose of this research is to have a better understanding of how AD progresses by identifying/detecting brain areas that degrade together during AD, and we can gain a better understanding of how the illness proceeds over the course of the a patient's life. The goal is to not only achieve diagnostic accuracy but also to provide relevant medical evidence. Thus, the primary objective of this work is to classify the degree of disease of the brain that undergoes neuronal degeneration concurrently with AD utilizing DL models and other ML algorithms. Consequently, hybrid techniques can indeed be developed by integrating the various strategies to enhance the system [19]. In this paper, a computer-aided design (CAD) system for AD classification has been made utilizing a CNN-SVM approach which is suggested as an improvised approach over the CNN model alone. The proposed CNN-SVM model includes convolutional layers (along with one additional fully connected layer) for extraction of features and then for classification SVM is used rather than the softmax or Sigmoid layers. Compared with traditional methods, the new method using hybrid CNN-SVM is directly driven by the data. Therefore, the proposed hybrid model in case of 2D MRI scans can also realize self-study of expression relations, which is considered an excellent for data representation of images. Further, CNN can independently learn and extract each local feature of data through multilayer convolution and pooling operations and obtain more effective abstract feature mapping than explicit feature extraction [20] methods. Additionally, SVM can help automatically learn the hierarchical feature representation of images which can be utilized based on the deep structure for effective binary as well as multiclass classification leading to reduction in the error rate of AD recognition. Thus, the improved system is divided into the tasks listed below:

- Conversion from NIfTI to 2D slices
- Selection of middle slices out of extracted slices for each subject
- Proposing of an enhanced CNN-SVM approach for extracting significant features and then classifying them

The developed CNN-SVM approach is then tested out versus the experimental end-to-end CNN model. As a consequence, utilizing SVM as a classifier at the end outperformed in comparison to utilizing softmax or Sigmoid function for classification.

The remaining part of the paper is structured as follows: Section 2 comprises a related work for AD classification, whereas Section 3 explores the theoretical framework of the CNN and SVM. Furthermore, Section 4 presents the details about dataset acquisition along with its preprocessing, as well as methodology adopted with its performance.  Section 5 outlines the research's conclusions and future scope.

## 2. Related Work

AD is a persistent and irreparable brains degenerative illness [21] that affects cognitive decline, depressive symptoms, linguistic confusion, decision-making process, and mental disability [22–24]. This disease also causes anatomical structures such as the hippocampus responsible for long-term memory and the cerebral cortex to shrink, while the ventricles in the brain expand. A healthcare professional can visualize disease progression based on these characteristics utilizing neuroimages of patients in the late stages of AD. Moreover, the intensity of each of these alterations in the nervous system varies with the severity of the disease, especially dramatic contraction of the hippocampi and cerebral cortex and ventricular enlargement visible clearly on neuroimaging at the final stages of the disease [25]. Thus, they suffer in the early stages of the disease often referred to as MCI [26], while not all MCI patients move to AD. MCI is a transitory phase from normal to AD where the person experiences minor changes in behavior that have been observable to the afflicted individuals along with close relatives. In such scenarios, the transition phase varies from around six months to three years, while one and a half year is the most usual. As a result, MCI participants usually split into 2 groups: convertible MCI and nonconvertible MCI [27]. Unfortunately, the underlying etiology of AD is still obscure to healthcare experts, and also no recognized treatments or remedies have been shown to avoid or reverse the development of AD [28]. Some of the ML and DL(CAD) based AD classification techniques will be discussed further below.

Scientists recently developed a variety of CAD diagnostic methods to support in disease diagnosis. As from 1970s till 1990s, experts established rule-based intelligent algorithms and afterwards supervised models. To build supervised algorithms, features were extracted from the clinical image data [29]. In view of the complex features of brain images, the researcher group of Han et al. in [30] proposed a DL-based methodology named as HCSAE (hierarchical convolutional sparse autoencoder) treated various CSAEs in an unsupervised hierarchy mechanism. The CSAEs retrieved the key aspects of the input utilizing the SAE and compiled the input data in a convolutional way that further enabled to derive impactful and accurate features and preserve plentiful complete details for brain imaging identification. Brain imaging fMRI data were used to validate their method, which demonstrated significant capability when compared to standard classifiers. The authors in [31] effectively differentiated AD fMRI data from healthy controls (HC) employing CNN and the well-known model LeNet-5. Additionally, they employed the LeNet model from Caffe DIGITS 0.2, which is inspired by Deep CNN. In their architecture, they deployed 2-CL layers along with a max-pooling layer after each CL. In the classification of AD vs. HC, the model obtained 96.9% overall accuracy. The experiment revealed that using CNN to capture stable features followed by DL classification has been the effective method for distinguishing diseased data from HC in fMRI. In [9], Gupta et al. evaluated filters or core retrieval using a sparse auto encoder. The authors evaluated it on different types of data: (a) MRI data and (b) natural images. Following the training of 100 bases which indicated lesions in MRI data, researchers deployed 2D convolutions to the MRI data. The Sigmoid activation function was then applied to derive feature activations. Subsampling max pooling was used to lessen the dimensions. Payan and Montana adopted the similar strategy to train a sparse autoencoder for feature extraction and then employed CNN on those learnt features. Similar to Gupta et al.'s model, the convolution layers were followed by subsampling pooling, a FC layer, and a softmax output layer with three outputs according to the class probabilities [32]. The researchers in [33] suggested the use of CNN in the diagnosis of AD, HC, and MCI. The authors particularly optimized VGGNet-16 for ternary classification of AD, MCI, and HC employing the AD Neuroimaging Initiative (ADNI) dataset. In contrast to other classifiers, they attained an overall accuracy of 92 percent. Another group of researchers in [34] recommended the AD classification model using a deep 3D CNN, which could also identify patterns and features identifying AD signs and adapting to varied application datasets. 3D-CNN was based on a 3D convolutional autoencoder which had previously been trained to detect structural form variations in sMRI. 3D CNN's top FC layers were then fine-tuned for each target-specific AD classification task. Research on the CADDementia MRI dataset without skull-stripping preprocessing revealed that 3D-CNN outperformed various classical models in terms of performance. The ADNI dataset was used to validate their model. The authors of [35] presented implementing a cascaded 3D-CNN in hierarchical manner to acquire nonlinear image characteristics that were ensemble for AD classification leveraging PET images of the brain. Initially, various deep 3D-CNNs are built on distinct local input image patches in ability to turn the local images into further concise strong features. Next, for classification purpose, a deep 3D CNN was developed to combine the high-level features. The proposed methodology enabled automatically grasping generalized features for identification given PET scans. Preprocessing the PET scans did not need any kind of registration and segmentation.  Table 1 illustrates the related studies on AD classification using various approaches.

Another group of researchers [43] attempted to address the challenge with a small set of medical data utilizing transfer learning, in which cutting-edge frameworks like VGG-16 and Inception-V4 (initialized with pretrained weights from the ImageNet dataset), and the FC layer was retrained with just a limited quantity of OASIS MRI neuroscans. Image entropy was also used to extract the most informative slices. Researchers proved the OASIS MRI dataset with training sizes nearly ten times lesser than the state-of-the-art, equivalent, or indeed higher accuracy could be obtained than existing DL-based techniques. Recently, DL models have been successfully applied to the Alzheimer's dataset to identify HC from other classes (MCI, cMCI, ncMCI, and AD).

## 3. Theoretical Background

### 3.1. Convolutional Neural Network

During the last decade, CNN has achieved ground breaking findings in a wide range of domains such as pattern recognition domains, from computer vision to speech classification [44, 45]. One of most advantageous element of CNNs is that they result in fewer of parameters in ANN. This success has motivated many academicians and research group authors to seek larger models required to perform complicated situations that were previously impossible with traditional ANNs; the far more significant hypothesis concerning CNN-solved issues is that they should not exhibit spatially dependent features [46]. In disease detection using medical data [47–49], researchers not need to concern regarding where the main features are in the image. Furthermore, the system is capable of capturing spatial-spectral correlations in MRI neuroscans [50], particularly if there is an occurrence of three-dimensional and 2-dimensional referring to medical image, via a process of minimization and potential optimization settings [51].

A standard CNN comprises of three primary layers: the convolutional layer (CL), the subpooling layer, and the fully connected (FC) layer [8, 52–54], illustrated in Figure 1. CNN's basic building component is the convolution operation. This performs the most of the computing load of the system. The layer computes the dot product of 2 matrices, one of which is the set of trainable parameters matrix known as a kernel or a filter and the other is the fraction of the input image. The product after convolution operation is thus evaluated as a 2D matrix, only with ultimate aim of every feature getting correlated to the summation of the elements of the kernel, and the image's sub cube. So, for an input with size *N*∗*N*∗*D*, where the *N*∗*N* is the height and width of image, *D* is the number of filters having spatial size of *F*, padding *P*, and stride *S*; designers can calculate the dimension of the output image using the below

(1) $$\begin{array}{c} N_{\text{out}}=\left[\frac{N-F+2\text{P}}{\text{S}}\right]+1. \end{array}$$

Afterwards, the pool operation replaces network output at specific places by generating a summarized score of adjacent outputs. One such contributes in minimizing the dimension of the feature or activations maps and therefore lowers the cost of calculation and weight involved. The pool operation is performed on each sliced of the representation separately. After the pooling operation, the size of image reduces as per

(2) $$\begin{array}{c} N_{\text{out}}=\left[\frac{N-F}{S}\right]+1. \end{array}$$

### 3.2. Support Vector Machine

SVMs are a fundamental aspect in learning concept. Algorithms are highly effective for a variety of tasks in engineering and science, notably classification concerns [55]. Inspired by Fisher's [56] classification techniques for splitting information, Boser et al. [57] proposed SVM polynomial kernel. SVM is the focus of considerable research since then, including deployments to a variety of relevant tasks, numerous modifications on the previous design, and some conceptual study. SVM tries to depict multidimensional data in a region partitioned by a hyperplane which isolates data elements into distinct classes. On new unseen data, the SVM as a classifier can reduce the classification error. SVM has been proven to be efficient for binary classification but inadequate for outlier noisy data.

## 4. Methodology and Implementation

### 4.1. Dataset Acquisition and Preprocessing

The dataset ADNI was included in this study. A list of all ADNI investigations may be found at http://adni.loni.usc.edu/wp-content/uploads/how to apply/ADNI Acknowledgement List.pdf [58]. This dataset was started in 2004 through National Institute on Aging (NIA), National Institute of Biomedical Imaging and Bioengineering (NIBIB) grants, and a variety of pharmaceutical industries and organizations. The prime focus of ADNI was to follow the status of early AD and MCI that used a blend of clinical and neuropsychological measures, MRI, fMRI, PET, and related biomarkers. The dataset accumulating document is maintained on the ADNI portal [59] which itself is directed by Michael W. Weiner, MD.

The dataset includes 50 participants from each of the three classes: CN, MCI, and AD as illustrated in Table 2. The 80% of the subjects were used for training and rest 20% utilized for testing the model. Each participant underwent approximately 3-4 MRI scans over the period of time. The dataset originally downloaded from site was available in the NIfTI format (3 dimensional). Firstly, we adopted Algorithm 1 as discussed below to convert an NIfTI extension files to 2D images (png format) since training a 3D CNN utilizing NIfTI files requires a long time and is relatively costly [60]. The count of recovered images (after conversion) corresponded to each of the single MRI scan was 256. Just the innermost 66 slices from a total of 256 were studied; the remaining (extreme side) was not considered since these exhibited no valuable features. Sample images extracted from NIfTI after conversion are shown in Figure 2.

### 4.2. Experimental Setup and Results Discussion

Figure 3 depicts the workflow for the proposed hybrid CNN-SVM architecture for AD classification which is divided into two stages: data collection and splitting of dataset, feature extraction and classification.  Figure 4 depicts the usage of CNN to extract features and SVM as a classifier on those derived features. This study's CNN architecture comprises of four convolutional layers which have a 160∗160 input image as input. 32 filters with kernel sizes of 3∗3 were chosen for the first and second CL. The third and fourth layers were each composed of 64 filters of the same size as the preceding one. All of the convolutional layers have the same padding and stride size of 2. The batch size of 32 with Adam optimizer, learning rate 0.0020, 128 dense units, and the ReLU activation function was adopted in all CL.

Just after feature extraction through CNN processes are completed, the SVM classifier is employed to classify ADNI images. SVM classifier training was carried out with feature maps encoded in matrix format. The training results were used to evaluate the ADNI test data. In fact, the automatically derived features from the CNN network were forwarded to the SVM component for training and testing on the ADNI dataset. The ADNI testing data is similarly preprocessed before being applied to test the classifier.

Table 3 demonstrates the overall impact of SVM as a classifier at the end versus end-to-end CNN for feature extraction and classification for train and test performance. Table 2 indicates that integrating SVM as a classifier on the derived features of CNN outperforms using CNN individually in both binary (AD vs. CN, CN vs. MCI, and AD vs. MCI) and ternary classification (CN vs. MCI vs. AD). The highest accuracy was recorded in the case of AD vs. CN binary classification, with 86.32 percent and 89.4 percent for the CNN and hybrid CNN-SVM models, respectively. In the case of ternary classification, the accuracy was 80.65 percent for CNN and 81.8 percent for the hybrid CNN-SVM model, respectively. There is a relative improvement (RI) of 3.57%, 1.78%, 0.8%, and 1.43% using the hybrid CNN-SVM model over the CNN model for AD vs. CN, CN vs. MCI, AD vs. MCI, and CN vs. MCI vs. AD for training accuracy. In contrast, the CNN-SVM model testing accuracy has a RI of 3.4%, 1.09%, 0.85%, and 2.83% higher than the CNN model.

In the case of binary classification, the accuracy of CN vs. MCI in the training sets is 83.71 percent and 85.2 percent, respectively, and for AD vs. MCI is 84.23 percent and 84.9 percent, which is lower than the accuracy of AD vs. CN. Furthermore, a significant comparison can be seen between classifications consisting of AD vs. MCI and CN vs. MCI with AD vs. CN, as it is harder to identify the early phase (i.e., MCI) from CN and AD.

### 4.3. Comparative Analysis with State-of-the-Art Datasets and Technologies

The availability of sufficient resources, as well as an imaging dataset, is critical to the creation of an AD classification system. However, in real-world applications, improved research in AD classification is now leading to a greater use of hybrid modeling approaches that are capable of achieving self-study of expressive correlations, which is regarded as an ideal method for visual data representation. The use of CNN for effective classification of MRI scans is similar to the more ordinary neural networks in that they are made up of hidden layers consisting of neurons with learnable parameters [23]. However, the earlier proposed methodologies by the researchers clearly lags automatically learning the hierarchical feature representation of images which otherwise can be utilized based on the deep structure for effective binary as well as multiclass classification [28, 44, 61].  Table 4 outlays a state-of-the-art comparison of diverse datasets and modeling methodologies, allowing for a relevant assessment of DL, transfer learning, and hybrid learning effectiveness.

## 5. Conclusion, Limitations, and Future Scope

### 5.1. Contribution of the Proposed Work

In addition to practical implications, the present study contributed to existing literature regarding AD. This study also contributed to the understanding of what kind of biomarkers could be utilized for AD and various techniques for classification of AD can be effectively utilized. The analysis of this study added to existing research by identifying a novel hybrid approach-based learning of the features that should be considered in early stages of the innovation process, compared to traditional methodologies of utilizing neural network which seems to be less important. This research further confirmed results of existing studies that emphasized the importance of modeling in detection of neurological diseases mainly AD and its availability of relevant resources [22, 29, 49, 62]. However, the present study also helped in the improved classification of the AD in comparison to our previously performed experimentations which in real-life world could contribute to an existing innovation and technology transfer literature and in biotechnology-focused studies. Moreover, the study contributed to prior theory by applying, validating, and extending a model for detection of AD. The results showed the improved performance of the multiclassification system using hybrid modeling CNN-SVM approach. Further, to strengthen the results, the study has been further experimented on the OASIS dataset keeping in mind the consideration of relevant biomarkers as well as applied a hybrid method approach. The management of AD in early stages process depends on the context and should be considered accordingly. In addition, existing research often utilized a standalone ML or DL technique for AD classification, hybrid modeling studies such that the present research contributed by linking two different methodologies (CNN and SVM). The study contributed to existing research by through hierarchical feature representation of images via CNN that can be well utilized for effective binary as well as multiclass classification through SVM which was often not done in prior studies in the domain of biomedical engineering and technology transfer.

### 5.2. Conclusion

AD is a progressive neurological condition in which brain cell loss causes in significant mental deterioration. It has been the most prominent type of dementia and also has a severely destructive influence on both the personal and sociocultural activities of individuals. Timely recognition of AD permits the sufferer to procure the optimal feasible medication. Various experts are investigating upon this issue, and yet many ways of recognizing AD have already been proposed. In this research, a CNN-SVM hybrid model for AD classification is proposed, which integrates automated feature extraction with CNN and classification with SVM. In order to identify AD, the network incorporates the strengths of CNN and SVM classifiers. The approach additionally prefers the adoption of automatically generated features versus hand-engineered features. Study results on the ADNI data for 50 subjects for each category CN, MCI, and AD suggested that a hybrid CNN-SVM using CNN for feature extraction and SVM for classification achieved a high accuracy for AD vs. CN binary classification with a RI of 3.4 percent for the testing dataset. The binary classification CN vs. MCI accuracy during the training set is 83.71 percent and 85.2 percent for CNN and Hybrid CNN-SVM model, respectively, while the accuracy of AD vs. MCI is 84.23 percent and 84.9 percent, which is lower than the accuracy of AD vs. CN. Additionally, a significant difference could be noticed between categories consisting of AD vs. MCI and CN vs. MCI with AD vs. CN, since it is more difficult to distinguish the early phase (i.e., MCI) from CN and AD.

### 5.3. Future Scope

The proposed hybrid modeling technique still has significant flaws. To begin, optimizing the parameters of the CNN alongside the implementation of SVM, such as the number of hidden layers, the size, and the number of kernels for each layer, is a difficult yet time-consuming operation. Furthermore, the proposed method's learnt characteristics lack adequate clinical information for visualization and interpretation of neurodegenerative disease AD. Nonetheless, in the near future, the aforementioned shortcomings will be overcome by configuring the CNN parameters based on optimum selection methodologies, employing an optimum kernel sizes, and effectively including the clinical features. Moreover, the authors chose a single MRI neuroimaging modality in this study since the integration of several other data modalities can give a comprehensive perspective of AD staging evaluation even further improve the model's performance. As a result, in the future, additional modalities, like as DTI and PET, might be employed in addition with MRI brain scans to identify AD and CN. Future applications of the suggested hybrid CNN-SVM include disease classification such as lung cancer, brain cancer detection, and autism detection.

## Figures and Tables

**Figure 1:** A typical CNN architecture.

**Figure 2:** Sample images extracted after conversion from NIfTI to png.

**Figure 3:** Flowchart of proposed hybrid CNN–SVM model.

**Figure 4:** Proposed hybrid CNN-SVM architecture.

**Algorithm 1:** NIfTI to png conversion

**Table 1:** Related work.

References	Year of reference	Techniques used	Main idea of the paper
[36]	2018	HadNet 3D-CNN	The researchers implemented a HadNet DL model to develop a classification system for MRI neuro-scans which was founded on a 3D CNN. The HadNet architecture's foundation comprised layered convolutions (inception methodology), that enabled additional internal features of the MRI scans relevant to AD. Additionally, HadNet's hyperparameters were fine-tuned using the Bayesian optimization procedure.
[37]	2019	3D-CNN	Researchers revealed numerous approaches for improving the performance of 3D CNN trained on sMRI neuroimaging dataset to identify classify AD. Authors further proved that instance normalization outperformed batch normalization, initial spatially downsampling reduced accuracy, broadening the framework provided stable improvements whereas extending depths did not, and finally including age as a feature input offered minor gain in performance.
[38]	2020	CNN-RNN-LSTM based	The authors concentrated on developing the three core models, which included CNN, long short-term memory (LSTM), and recurrent neural networks (RNN), and long short-term memory (LSTM) in the initial phase. The ensemble approach was then applied in the next step to integrate all three models adopting a weighted mean strategy. Bagging was applied in all three approaches to reduce variability. Thus, three bagged models were integrated with the ensemble technique.
[39]	2021	VGG, ResNet-50, AlexNet	This study is aimed at identifying MRIs of AD patients into several classes via various transfer learning models such as VGG16, ResNet-50, and AlexNet, along with CNN.
[40]	2020	3D ResNet-18	A technique by using transfer learning in 3D CNNs that enables learning to be transferred from 2D image datasets to 3D image datasets was suggested by the authors.
[41]	2021	2D-CNN	With parameter optimization a 2D-CNN was employed to assess architectural impact in improving the diagnostic accuracy of four classes of images—mild, very mild, moderate, and nondemented considering AD.
[42]	2022	Sliding window association test- (SWAT-) CNN	SWAT-CNN: a three-step approach presented by researchers for detecting biological variants that leverages DL technique to determine phenotypic expression single-nucleotide polymorphisms that may be utilized to build appropriate AD classifier.

**Table 2:** Splitting of dataset into training and testing.

Subject or participant type	Total no of subjects	No of subjects (training)	No of MRI scans (NIfTI files)	No of images extracted	Total used images	No of subjects (testing)	No of MRI scans (NIfTI files)	No of images extracted	Total used images
CN	50	40	144	36,864	9,504	10	33	8,448	2,178
MCI			104	26,624	6,864		32	8,192	2,112
AD			111	28,416	7,326		33	8,448	2,178

**Table 3:** Comparison of CNN and hybrid CNN-SVM model training and testing accuracy.

Classification	Accuracy (%) CNN model		Accuracy (%) hybrid CNN-SVM model	
	Training	Testing	Training	Testing
AD vs. CN	86.32	85.1	89.4	88
CN vs. MCI	83.71	82.9	85.2	83.8
AD vs. MCI	84.23	82.4	84.9	83.1
CN vs. MCI vs. AD	80.65	78.1	81.8	80.3

**Table 4:** Comparative analysis of the proposed approach with previously proposed state-of-the-art classification systems.

References	Year of reference	Dataset details	Modeling techniques	Classification accuracy (%)	Summary
[62]	2019	ADNI	DL-based method	86	The researchers extracted significant features from structural MRI imaging recorded at the baseline clinical visit using a parameter-efficient deep CNN architecture inspired by clustered and segmented convolutions.
[63]	2018	ADNI	Transfer learning from CNN	67.6	The research team used scraped pretrained or trained AlexNet CNN as a generalized feature representation of a 2D MRI neuroimaging, wherein dimensionality was compressed through PCA+TSNE before classification using a basic ML technique.
[64]	2019	ADNI	KNN	43.3	Six different ML and data mining methods have been applied to the ADNI dataset in classifying the five distinct phases of the AD and determine one of most unique feature for each AD's phase.
			Decision tree	74.2	
			Rule reduction	69.7	
			Naïve Bayes	74.7	
			Generalized linear model	88.24	
			DL	78.23	
[65]	2019	ADNI	Convolutional autoencoder (CAE)	86.6	The investigators applied unsupervised learning focused on CAE to address classification challenge for AD/NC and supervised pretrained models to tackle the pMCI/sMCI classification task. A gradient-based visualization technique which resembles the temporal impact of the CNN designer's choice has been implemented to find the most relevant biomarkers associated to pMCI and AD.
[66]	2020	ADNI	VGG variant CNN	73.4	The researchers minimized information loss when splitting 3D volume MRI brain scans into 2D images, the authors used 3D models and analyzed data with 2D convolutional filters.
		OASIS		69.9	
[67]	2021	ADNI	VGGNet	83.7	During developing the DL network, the methods involved a huge volume of labeled data. To diagnose the initial phases of AD, experts exploited layer-wise transfer learning as well as tissue segmentation of MRI scans. Researchers deployed the VGG model family containing pretrained weights of ImageNet data.
Proposed methodology	—	ADNI	Hybrid CNN-SVM	88	This research presented a new adaptive model based on CNN and SVM, incorporating the strengths of CNN in feature extraction and SVM in classification; to create a hybrid CNN-SVM model for classify AD using the MRI ADNI dataset.
		OASIS		86.2	

## Data Availability

The data that support the findings of this investigation are available from ADNI (http://adni.loni.usc.edu); however, they are subject to restrictions because they were utilized under permissions for this work and are therefore not publicly available. The authors' data are, however, available upon reasonable request and with ADNI's approval.
